This article has been retracted.

# MicroRNA-497 inhibits thyroid cancer tumor growth and invasion by suppressing BDNF

**DOI:** 10.18632/oncotarget.13747

**Published:** 2016-12-01

**Authors:** Peisong Wang, Xianying Meng, Yan Huang, Zhi Lv, Jia Liu, Guimin Wang, Wei Meng, Shuai Xue, Qiang Zhang, Pengju Zhang, Guang Chen

**Affiliations:** ^1^ Department of Thyroid Surgery, The First Hospital of Jilin University, Chaoyang District, Changchun 130021, China; ^2^ Department of Orthopaedic Surgery, China-Japan Union Hospital of Jilin University, Jingyue District, Changchun 130033, China; ^3^ Jilin Academy of Agricultural Sciences, Nanguan District, Changchun 130000, China

**Keywords:** miR-497, thyroid cancer, BDNF, tumorigenesis, metastasis

## Abstract

miR-497 reportedly plays critical roles in tumor development and progression in many types of cancers. We therefore investigated the function and underlying mechanism of miR-497 in thyroid cancer. We found that miR-497 is downregulated in thyroid cancer tissues, and that miR-497 levels are negatively correlated with advanced clinical stage and lymph node metastasis. Overexpressed miR-497 suppressed thyroid cancer cell proliferation, colony formation, migration, and invasion *in vitro*, and inhibited tumorigenesis *in vivo*. Moreover, brain-derived neurotrophic factor (BDNF), a known oncogene, was confirmed as a direct target of miR-497 in thyroid cancer cells. miR-497 overexpression suppressed BDNF expression and its downstream pathway(PI3K/AKT)*in vitro* and *in vivo*. BDNF levels were upregulated and inversely correlated with miR-497 levels in human thyroid cancer specimens. Rescue experiments showed that forced overexpression of BDNF effectively reversed the tumor suppressive functions of miR-497. These results show that miR-497 is a thyroid cancer tumor suppressor that acts by repressing BDNF.

## INTRODUCTION

Thyroid cancer is the most common endocrine malignancy, and is one of the most rapidly growing in many countries over the last several decades [1]. Despite advanced diagnostic and therapeutic approaches that have greatly improved long-term survival from thyroid cancer, a significant proportion of patients exhibit locoregional recurrence or distant metastases within 10 years [2, 3]. Better understanding of the molecular mechanisms underlying carcinogenesis and progression in thyroid cancer would contribute to finding novel diagnosis markers and novel therapeutic targets.

MicroRNAs (miRNAs) are a class of endogenous, small, non-coding RNAs. They regulate posttranscriptional gene expression by binding to the 3′-untranslated region (UTR) of target mRNAs, leading to target mRNA cleavage or translation inhibition [4]. miRNAs regulate diverse biological processes, such as cell proliferation, cell cycle, apoptosis, migration, invasion, and differentiation [5, 6]. miRNAs also affect cancer development and progression, and can serve as oncogenes or tumor suppressors [7–9]. Specifically, miRNAs are involved in thyroid cancer tumorigenesis [10, 11], suggesting that miRNAs could act as potent therapeutic targets or diagnosis markers for thyroid cancer.

miR-497, a highly conserved miRNA encoded by the first intron of the MIR497HG (Gene ID: 100506755) gene on human chromosome 17p13.1 [12], is a tumor suppressor in multiple cancers [13–19]. The aim of this study was to investigate the discrete role and molecular mechanism of miR-497 in thyroid cancer.

## RESULTS

### miR-497 is downregulated in human thyroid cancer specimens

To determine miR-497 levels in human thyroid cancer specimens, qRT-PCR analysis was performed in 48 pairs of thyroid cancer tumor specimens and matched adjacent normal tissues. Levels of miR-497 in thyroid cancer tissues were downregulated compared to adjacent normal tissues (Figure 1A). To further investigate the clinicopathological significance of miR-497 level in patients with thyroid cancer, 48 patients were divided into 2 subgroups based on mean (0.312) of all thyroid cancer samples: low miR-497 group (< 0.312, 27 cases) and a high miR-497 group (> 0.312, 21 cases). We found that miR-497 levels in tumor tissues were correlated with clinical stages and lymph node metastasis, but not with age, gender, or tumor size (Table 1). In advanced clinical stages (TNM stage III-IV),miR-497 levels were downregulated compared with those in low clinical stages(TNM stage I and II) (Figure 1B). Moreover, miR-497 levels were decreased in the patients with lymph node metastases compared to the patients without lymph node metastases (Figure 1C).

**Figure 1:** miR-497 expression is downregulated in human thyroid cancer tissues (**A**) Relative miR-497 levels were determined in 48 pairs of thyroid cancer specimens and corresponding adjacent normal tissues. U6 RNA levels were used as an internal control. (**B**) Relative miR-497 levels in different clinical stages of thyroid cancer tissues. U6 RNA levels were used as an internal control. (**C**) Relative miR-497 levels in thyroid cancer with/without lymph node metastasis. *p < 0.05, **p < 0.01.

**Table 1:** Association between miR-497 expression and clinicopathological features of human thyroid cancer

Variables	No. of cases	miR-497 expression		*p* value
		Low (*n*%)	High (*n*%)	
Age(years)				*p* > 0.05
< 50	23	13 (56.5)	10 (43.5)	
≥ 50	25	14 (56.0)	11 (44.0)	
Gender				*p* > 0.05
Male	19	10 (52.6)	9 (47.4)	
Female	29	17 (58.6)	12 (41.4)	
TNM stage				*p* < 0.01
I-II	31	12 (38.7)	19 (61.3)	
III-IV	17	15 (88.2)	2 (11.8)	
Tumor size				*p* > 0.05
< 5 cm	30	18 (60.0)	12 (40.0)	
≥ 5 cm	18	9 (50.0)	9 (50.0)	
Lymph node metastasis				*p* < 0.01
No	33	13 (39.4)	20 (60.6)	
Yes	15	14 (93.3)	1 (6.7)	

### miR-497 inhibits thyroid cancer cell proliferation, migration, and invasion

To examine the role of miR-497 in thyroid cancer development, TPC-1 cells with low miR-497 expression were transfected with miR-497 mimic or miR-Negative Control (miR-NC). qRT-PCR analysis confirmed that miR-497 expression was upregulated in cells transfected with miR-497 mimic compared to cells transfected with miR-NC (Figure 2A). MTT, colony formation, wound healing, and transwell invasion assays were performed in TPC-1 cells transfected with miR-497 mimic or miR-NC. We found that miR-497 overexpression inhibited cell proliferation, colony formation, migration, and invasion of TPC-1 cells (Figure 2B–2E). These results suggested that miR-497 acts as a tumor suppressor in thyroid cancer cells.

**Figure 2:** miR-497 inhibits cell proliferation, colony formation, migration and invasion of thyroid cancer cells (**A**) Relative miR-497 levels were measured in TPC-1 cells transfected with miR-497 mimic or miR-NC by qRT-PCR. U6 RNA levels were used as an internal control. (**B**–**E**) Cell proliferation, colony formation, migration, and invasion were determined in TPC-1 cells transfected with miR-497 mimic or miR-NC. *p < 0.05, **p < 0.01.

### BDNF is directly suppressed by miR-497 in thyroid cancers cells

To fully understand the mechanism of miR-497 in inhibiting human thyroid cancer progression, three bioinformatic databases (TargetScan, miRanda, and PicTar) were used to predict miR-497 targets. Focusing on genes that promoted tumor progression and metastasis, BDNF was selected as a putative miR-497 target based on a sequence at 300–306 bp (Figure 3A). To explore whether miR-497 targets BDNF by binding to its 3′-UTR region, TPC-1 cells were co-transfected with the wild type (WT) or mutant-type (MUT) BDNF luciferase reporter plasmid, and miR-497 mimic or miR-NC. After 48 h transfection, the luciferase activities in these cells were measured. Luciferase activities were reduced in the cells cotransfected with the WT-BDNF reporter plasmid and miR-497 mimic, but not in the cells cotransfected with the MUT-BDNF reporter plasmid and miR-497 mimic (Figure 3B). Forced expression of miR-497 decreased BDNF expression on both the mRNA level and protein level (Figure 3C, 3D). In addition, miR-497 overexpression also decreased p-PI3K and p-AKT expression, which are known downstream molecules of BDNF (Figure 3D). These results suggested that miR-497 directly suppresses BDNF by binding its seed region of the 3′-UTR region in human thyroid cancer cells.

**Figure 3:** BDNF is directly suppressed by miR-497 in thyroid cancer cells (**A**) The complementary pairings of miR-497 with BDNF wild-type (WT) and mutant (MUT) 3′-UTR reporter constructs. (**B**) Relative luciferase activity in TPC-1 cells co-transfected with WT or MUT 3′-UTR BDNF reporter plasmids and miR-497 or miR-NC. WT: wide-type; MUT: mutant-type. (**C**) BDNF mRNA levels were determined in TPC-1 cells transfected with miR-497 or miR-NC. β-actin was used as the internal control. (**D**) The BDNF, PI3K, p-PI3K, AKT, and p-AKT protein levels were determined in TPC-1 cells transfected with miR-497 or miR-NC. GAPDH was used as the internal control. *p < 0.05, **p < 0.01.

### BDNF has an inverse correlation with miR-497 expression in thyroid cancer

We measured BDNF mRNA and protein levels in thyroid cancer tissues and the corresponding adjacent normal tissues by qRT-PCR and immunohistochemistry. Our results showed that both BDNF mRNA and BDNF protein levels were increased in the thyroid cancer tissues compared to the adjacent normal tissues (Figure 4A, 4B). Next, we determined the correlation between BDNF mRNA levels and miR-497 expression in the same human thyroid cancer specimens using Spearman's rank correlation analysis. The expression of miR-497 was inversely correlated with BDNF mRNA levels in the 48 patients with thyroid cancer (r = −0.651; *p* < 0.001) (Figure 4C).

**Figure 4:** BDNF expressionis upregulated, and inversely correlated with miR-497 expression in NSCLC tissues (**A**) BNDF mRNA expression in 48 cases of thyroid cancer tissue and adjacent normal tissues were detected by qRT-PCR. β-actin was used as an internal control. (**B**) BDNF protein expression was detected in thyroid cancer tissue and adjacent normal tissues by immunohistochemistry. (**C**) Spearman's correlation analysis was used to determine the correlations between the levels of BDNF and miR-497 in human thyroid cancer (*n* = 48). *p < 0.05, **p < 0.01.

### Restoration of BDNF reverses miR-497-suppressed cell proliferation, colony formation, migration, and invasion of thyroid cancer cells

To test the functional relevance of miR-497 suppressing BDNF in thyroid cancer, we generated a BDNF overexpressing vector, and transfected it into TPC-1 cells. Forced expression of BDNF rescued miR-497-suppressed BDNF expression on the mRNA level and protein level (Figure 5A, 5B). Importantly, forced expression of BDNF also restored miR-497-inhibited cell proliferation, colony formation, migration, and invasion of thyroid cancer cells (Figure 5C–5F). These results suggest miR-497 inhibits thyroid cancer by repressing BDNF.

**Figure 5:** Restoration of BDNF reversed the tumor suppressive effect of miR-497 in thyroid cancer (**A**, **B**) BDNF expression on mRNA level (A) and protein level(B) was determined in TPC-1 cells transfected with miR-497 mimic with/without BDNF overexpression plasmid. (**C**–**F**) Cell proliferation, colony formation, migration, and invasion were determined in TPC-1 cells transfected with miR-497 mimic with/without BDNF overexpression plasmid.*p < 0.05, **p < 0.01.

### miR-497inhibits thyroid cancer tumorigenicity *in vivo* by suppressing BDNF

To examine miR-497's role in thyroid cancer tumorigenicity *in vivo*, TPC-1 cells transfected with miR-497 mimic or miR-NC were harvested, and then injected into nude mice. The resulting tumors were measured in size 15 days after injection. Tumor growth was lower in the miR-497 group from Day 20 to Day 35 than that of the miR-NC group (Figure 6A). Mice were sacrificed 35 days after injection, and tumor tissues were striped and weighed. The miR-497 overexpression group displayed smaller size and lower weight tumors than that of the miR-NC group (Figure 6B, 6C).

**Figure 6:** miR-497 suppresses thyroid cancer tumorigenicity in vivo by repressing BDNF (**A**) Growth curves for tumor volumes in xenografts of nude mice from the TPC-1/miR-497 and TPC-1/miR-NC groups. (**B**) Representative images of tumors from the TPC-1/miR-497 and TPC-1/miR-NC groups. (**C**) Weights of tumors from the TPC-1/miR-497 and TPC-1/miR-NC groups. (**D**) Relative miR-497 levels were determined in tumor tissues from TPC-1/miR-497 and TPC-1/miR-NC groups by qRT-PCR. U6 RNA levels were used as an internal control. (**E**) BDNF mRNA levels were determined in tumor tissues from TPC-1/miR-497 and TPC-1/miR-NC groups by qRT-PCR. β-actin was used as the internal control. (**F**) The BDNF, PI3K, p-PI3K, AKT, and p-AKT protein were measured in tumor tissues from TPC-1/miR-497 and TPC-1/miR-NC groups by Western blot. GAPDH was used as the internal control. *p < 0.05, **p < 0.01.

We also determined miR-497 and BDNF levels in the tumor tissues. miR-497 expression was increased in the miR-497 group compared to the miR-NC group (Figure 6D), while BDNF mRNA and protein levels were decreased (Figure 6E, 6F). We also found that levels of p-PI3K and p-AKT in tumor tissues from the miR-497 overexpression group were decreased compared to the miR-NC group (Figure 6F). These data indicate that miR-497 suppresses thyroid cancer tumorigenicity *in vivo* by repressing BDNF.

## DISCUSSION

miR-497, a member of the miR-15 family (miR-15a, miR-15b, miR-16–1/2, miR-195, miR-424 and miR-497), has been reported to be downregulated, and function as a tumor suppressor, in many types of cancers [13–19]. However, recently two reports reveal that miR-497 expression is upregulated, and functions as an oncogene, in glioma [20] and colorectal cancer [21]. These inconsistent findings indicate that dysregulation of miR-497 may play diverse roles in different cancers depending on the detail tumor type and the cellular microenvironment [22]. Here, we found that miR-497 expression was downregulated in thyroid cancer samples compared with adjacent normal tissues. miR-497 expression was negatively associated with advanced clinical stage and lymph node metastasis. Restoration expression of miR-497 significantly inhibited cell proliferation, colony formation, migration, invasion, and suppressed tumor growth in nude mice. These results suggested that miR-497 inhibits tumorigenicity in thyroid cancer.

miRNAs bind to the 3′-UTR of a target gene to regulate its expression to exert its biological function[6]. To identify the target genes of miR-497, three bioinformatic databases (TargetScan, miRanda, and PicTar) were used to predict gene targets for miR-497. Brain-derived neurotrophic factor (BDNF) was selected as a target gene due to its known role in promoting tumorigenesis and cancer progression [23–27]. BDNF, a member of the neurotrophin family, is also involved in the development and regeneration of neurons [28]. BDNF can also bind to its major receptor, tropomyosin-related receptor kinase B (TrkB), leading to the activations of multiple downstream signal pathways, such as PI3K/AKT, RAS/ERK, PLC/PKC, AMPK/ACC, and JAK/STAT pathways [29], which promote tumorigenesis. Specifically, PI3K/AKT pathway has been widely reported to be involved in thyroid cancer progression and development [30, 31]. Several miRNAs, such as miR-107 [32], miR-15a-5p [33], miR-204 [34], and miR-206 [35], inhibit cancer progression by suppressing BDNF.

Here, we confirmed that BDNF is suppressed by miR-497 in thyroid cancer by luciferase activity assay, qRT-PCR, and western blot. We also found that miR-497 overexpression could inhibit BDNF expression, and inhibited its downstream signal pathways (PI3K/AKT) *in vitro* and *in vivo*. Moreover, BDNF expression was upregulated, and inversely correlated with miR-497 in thyroid cancer tissues. Restoration of BDNF effectively reversed the tumor-suppressive functions of miR-497 on thyroid cancer cell proliferation, colony formation, migration, and invasion. These results show that miR-497 inhibits thyroid cancer by suppressing BDNF, suggesting that miR-497 is a potential therapeutic target for thyroid cancer.

## MATERIALS AND METHODS

### Clinical specimens

Human thyroid cancer specimens and adjacent normal tissues (48 pairs) were obtained from patients who underwent surgical resection in the Department of Thyroid Surgery, the First Hospital of Jilin University (Changchun, China). All tissue samples were snap-frozen in liquid nitrogen immediately after surgery, and stored in liquid nitrogen until use. All samples were histologically classified by two clinical pathologists (Changchun, China). The experiment protocols were approved by the ethics committee of Jilin University (Changchun, China), and all patients signed a written informed consent form.

### Cell culture and transfection

The human thyroid cell line TPC-1 was purchased from the Type Culture Collection of the Chinese Academy of Sciences (Shanghai, China), and were grown in DMEM medium (Gibco BRL, USA) at 37°C in a 5% CO_2_ incubator. The medium was supplemented with 10% fetal bovine serum (Gibco BRL), 100 units of penicillin/ml, and 100 ng of streptomycin/ml.

The TPC-1 cells were plated in 6-well plates at a density of 30,000 cells/ml. After being grown to 70~80% confluence, cells were transfected with miR-497 mimic (UGUUUGGUGUCACACGACGAC) (Gene Pharma Co., Ltd., Shanghai, China) or negative control (miR-NC,UUCUCGAACGUGUCACGUUUU) using Lipo fectamine 3000 (Invitrogen, CA, USA) at a final concentration of 100 nM. For BDNF overexpression, the open reading frame (ORF) coding BDNF was amplified by PCR, and cloned into pcDNA3.1 plasmid(Invitrogen). The transfection was conducted using Lipofectamine 3000 per manufacturer's instructions.

### Total RNA extraction, reverse transcription, PCR, and quantitative real time-PCR

Total RNA was isolated from cultured cells or tissues using Trizol reagent (Invitrogen), per the manufacturer's instructions. miR-497 expression was detected using the TaqMan MicroRNA assay Kit (Applied Biosystems, Foster City, CA, USA), with an ABI7900 real-time PCR system (Applied Biosystems), using miR-497 and U6 primers (Applied Biosystems). To determine BDNF mRNA levels, total RNAs was reversely transcribed into cDNA using RT Reagent Kit (Takara, Dalian, China)with oligo-dT primers. The quantitative PCR assay was performed using the Real-time PCR Mixture Reagent (Takara), with a ABI7900 real-time PCR system, using the specific primers of BDNF and β-actin as previously described [27]. The relative miR-497 levels or BDNF mRNA levels were quantified by measuring cycle threshold (Ct) values, and normalized using the 2^–ΔΔCt^ method relative to U6 or β-actin, respectively.

### Cell proliferation and colony formation assays

Cell proliferation was determined using the MTT assay (Sigma, USA). Transfected cells were seeded to 96-well plates, at approximately 5,000 cells per well, and maintained in DMEM medium for 24 h- 72 h. At the indicated time (24 h, 48 h, and 72 h), 100μl of spent medium was replaced with an equal volume of fresh medium containing 0.5 mg/ml MTT(Sigma), and incubated at 37°C for 4 h. The 150 μl of DMSO (Sigma) were added to each well for 10 min. The absorbance at 490 nm was measured with a microplate spectrophotometer (Bio-Tek Instruments Inc., Winooski, VT, USA).

For the colony formation assay, transfected cells were seeded into six-well plates at 500 cells per well, and cultured for 14 days. Cells were washed twice with PBS, fixed with 4% paraformaldehyde for 20 min, and then stained with 1% crystal violet (Sigma). The number of colonies formed was counted in five randomly selected fields under a light microscope (Olympus, Tokyo, Japan).

### Cell migration and invasion assays

To examine the migration ability of cells *in vitro*, a wound-healing assay was performed. Transfected cells were seeded in 6-well plates, and grown to 90% confluence. Afterwards, artificial wounds were created by 200 μl pipette tips. After wounding, the medium was changed to fresh, serum-free medium to remove cellular debris. Wound healing was observed and photographed at different time points (0 and 24 h) using a light microscope (Olympus).

Cell invasion was determined using a Transwell chamber with a pore size of 8μm, and the inserts were precoated with Matrigel (BD Bioscience, San Jose, CA, USA). The 2 × 10^4^ transfected cells were added to upper transwell chambers in serum-free medium. The lower chamber was filled with 600 μl of the medium, containing 10% FBS as the nutritional attraction. After incubation for 48 h in a humidified atmosphere of 5% CO2 at 37°C, noninvading cells were removed from the top well with a cotton swab. Invasive cells that attached to the lower surface of the membrane insert were fixed in 90% alcohol, stained with 0.1% crystal violet for 5 min, and then photographed under a light microscope (Olympus). The number of invaded cells was counted in five randomly selected fields.

### Dual-luciferase reporter assay

For the dual-luciferase assay, 3′-untranslated region (3′-UTR) regions of BDNF containing predicted miR-497 seed-matching sites and corresponding mutant sites were amplified by PCR using human cDNA template. They were then inserted downstream of the firefly luciferase gene in a pGL3-promoter vector (Ambion, Austin, TX, USA) at the NheI and XhoI restriction sites. These constructs were validated by DNA sequencing. TPC-1 cells were seeded in a 24-well plate and co-transfected with wild-type(WT) or mutant-type(MUT) 3′-UTR of BDNF reported plasmid, miR-497 mimic or miR-NC, and pRL-TK plasmid. Luciferase activities in the cells were determined 48 h after transfection using the Dual LuciferaseReporter Assay System (Promega, WI, USA), per the manufacturer's recommendations.

### Western blotting

Tissue samples or cultured cells were lysed with RIPA peptide lysis buffer (Beyotime Biotechnology, Jiangsu, China) containing 1% protease inhibitors (Pierce, Rockford, IL, USA). The total protein concentration was determined by a BCA kit (Pierce). Total protein(30μg) from each sample were electrophoresed on 10% sodium dodecyl sulfate polyacrylamide gel electrophoresis (SDS-PAGE), and transferred onto nitrocellulose membranes (Santa Cruz Biotechnology, Inc, USA). After blocked in 5% nonfat milk, the membranes were probed with the primary antibodies overnight at 4°C, and then with the corresponding secondary antibodies conjugated to horseradish peroxidase (HRP, Santa Cruz Biotechnology). Band signals were visualized using an enhanced chemiluminescence kit (Pierce, Minneapolis, MN, USA). Primary antibodies were used as follows: anti-BDNF (1:1000, Santa Cruz Biotechnology), anti-PI3K (1;1000, Cell Signaling Technology, USA),anti-p-PI3K (1;1000, Cell Signaling Technology), anti-AKT (1;1000, Cell Signaling Technology), anti-p-AKT (1:800, Cell Signaling Technology), and anti-GAPDH (1:3000, Santa Cruz Biotechnology). GAPDH was used as an internal control.

### Immunohistochemistry

Immunohistochemistry was performed using the SP method (Ultra Sensitive TM-SP) per manufacturer's instructions. Tissue sections from thyroid cancer and normal thyroid tissues were deparaffinized, and treatedwith methanol that contained 3% hydrogen peroxide for 30 min. Sections were then incubated with the primary antibody against BDNF (1:400, Santa Cruz Biotechnology) overnight at 4 °C. After incubation with biotin-conjugated secondary antibody for 10 min at room temperature, streptavidin-peroxidase was added for 10 min at room temperature. Sections were then treated with freshly prepared DAB solution for 5min. The slides were counterstained with hematoxylinand mounted.

### *In vivo* tumorigenesis assay

Ten male nude mice (BALB/c-null, 6-week-old, 18–20 g) were purchased from the Laboratory Animal Center of Jilin University (Changchun, China), and bred in special pathogen-free (SPF) conditions. All animal procedures were performed in accordance with Institutional Animal Care and Use Committee guidelines of Jilin University (Changchun, China).

2 × 10^6^ TPC-1 cells transfected with miR-497 mimic or miR-NC were harvested, washed, and re-suspended in 100 μl of serum-free DMEM medium. The cells were then injected subcutaneously into each side of the posterior flank of each nude mouse. Tumor sizes were measured every five days from the 15^th^ day of injection. Tumor volume was monitored and calculated according to the formula: V = 0.5 ×L (length) × W^2^ (width) by measuring tumor length and width using vernier calipers. Mice were sacrificed 35 days after injection, and tumor tissues were dissected and weighed. miR-497 and BDNF and its downstream protein expression were determined in tumor tissues by qRT-PCR and western blot, respectively.

### Statistical analysis

Statistical analysis was performed using the by Statistical SPSS Version 19.0 (IBM, Chicago, USA). All data were presented as the mean ± SD (standard deviation) of at least three independent experiments. A student's *t* test was used to compare the difference between two groups. One-way ANOVA was used to examine the difference among more than two groups. The correlations between miR-497 levels and BDNF mRNA levels were analyzed using Spearman's rank test. The differences were considered significant at *p* < 0.05.
